# Transdermal agomelatine microemulsion gel: pyramidal screening, statistical optimization and *in vivo* bioavailability

**DOI:** 10.1080/10717544.2017.1365392

**Published:** 2017-08-23

**Authors:** Mayada Said, Ibrahim Elsayed, Ahmed A. Aboelwafa, Ahmed H. Elshafeey

**Affiliations:** Department of Pharmaceutics and Industrial Pharmacy, Faculty of Pharmacy, Cairo University, Cairo, Egypt

**Keywords:** Microemulsion, transdermal, D-optimal mixture design, optimization, agomelatine

## Abstract

Agomelatine is a new antidepressant having very low oral drug bioavailability less than 5% due to being liable to extensive hepatic 1st pass effect. This study aimed to deliver agomelatine by transdermal route through formulation and optimization of microemulsion gel. Pyramidal screening was performed to select the most suitable ingredients combinations and then, the design expert software was utilized to optimize the microemulsion formulations. The independent variables of the employed mixture design were the percentages of capryol 90 as an oily phase (X_1_), Cremophor RH40 and Transcutol HP in a ratio of (1:2) as surfactant/cosurfactant mixture ‘S_mix_’ (X_2_) and water (X_3_). The dependent variables were globule size, optical clarity, cumulative amount permeated after 1 and 24 h, respectively (Q1 and Q_24_) and enhancement ratio (ER). The optimized formula was composed of 5% oil, 45% S_mix_ and 50% water. The optimized microemulsion formula was converted into carbopol-based gel to improve its retention on the skin. It enhanced the drug permeation through rat skin with an enhancement ratio of 37.30 when compared to the drug hydrogel. The optimum ME gel formula was found to have significantly higher C_max_, AUC _0–24 h_ and AUC_0–∞_ than that of the reference agomelatine hydrogel and oral solution. This could reveal the prosperity of the optimized microemulsion gel formula to augment the transdermal bioavailability of agomelatine.

## Introduction

Major depressive disorder (MDD) is a kind of depression characterized by a persistent severe depressed mood for most of time for a two-week period or more (Andrews et al., 2005). It causes disability and interfering with the ability to eat, sleep, study and work (Dempster et al., 2014; Du et al., 2015). Selective serotonin reuptake inhibitors (SSRI), the first choice for the treatment of depression, act by inhibiting the presynaptic reuptake of serotonin thus increasing the free serotonin available to bind to postsynaptic receptors (Preskorn, 1997; Ban, 2001).

Agomelatine is a novel drug acting as an agonist to the melatonergic receptors and antagonist to the serotonergic 5-HT_2c_ receptors (Millan et al., 2003). The recommended dose of agomelatine is 25 mg once daily taken at bedtime. During its development, agomelatine showed high safety profile and tolerability. This could be related to its novel mechanism of action that avoids the systemic serotonin release (Loo et al., 2002; Kennedy & Emsley, 2006; Montgomery, 2006; Rouillon, 2006). Agomelatine is well and rapidly absorbed after oral administration (80%) but it has low absolute bioavailability (less than 5%) due to extensive first pass metabolism (Zupancic & Guilleminault, 2006; Anurag et al., 2010).

Transdermal drug delivery system increases patient compliance, avoids gastrointestinal irritations, reduces first pass metabolism of drugs, sustains drug action and reduces side effects. So, there are many researches in recent years about it (McNeill et al., 1992; Azeem et al., 2009a). The stratum corneum restricts the transport of most drugs through the skin and considered as a main obstacle against drug permeation. Therefore, various techniques are used to enhance transdermal drug permeation, including the use of nanocarriers (e.g. microemulsions, nanoparticles and liposomes), penetration enhancers and physical techniques, such as iontophoresis, microneedles and electroporation, alone or in combination with other method (Essa et al., 2004; Wang et al., 2007; Balaguer-Fernandez et al., 2010; Vaghani et al., 2010; Nair et al., 2011). Drug carriers, such as microemulsions, nanoparticles and liposomes are a common and useful for transdermal drug delivery as they can alter the physical characteristics of applied drug and increases its transport across the skin (Nicoli et al., 2001; Lee & Langer, 2003; Essa et al., 2004; Liu et al., 2008; Xing et al., 2009; Tsai et al., 2010).

Microemulsions (ME) are thermodynamically stable and optically isotropic systems consisting of oil, water, surfactants and cosurfactant. They are thermodynamically stable and easily manufactured. Moreover, they enhance drugs solubility and permeability (Lehmann et al., 2001; Wu et al., 2001; Paolino et al., 2002; Peltola et al., 2003; Yuan et al., 2006; Spernath et al., 2007; Liu et al., 2008; Tsai et al., 2010). D-optimal mixture design was found to be the most suitable for microemulsion systems when compared to other designs as microemulsions are composed of three components which are oil, S_mix_ and water. Moreover, the use of D-optimal design facilitated setting different constraints for different factors where the sum of all components is constant (i.e.100% w/w) (Barot et al., 2012).

The aim of this study was to develop an optimized ME formula able to overcome the shortcomings of the oral agomelatine delivery. Pyramidal screening was adopted to select the most suitable oil, surfactant and cosurfactant. This technique was found to be superior over the discrete screening, which depends on the drug solubility in each individual component, in the aspect of considering the power of the used surfactant and cosurfactant to emulsify the incorporated oil (Azeem et al., 2009b). After screening and selection of formulation components, D-optimal mixture design was utilized to statistically optimize agomelatine loaded MEs. The optimized ME dispersion had been designed to be transformed into gel and then, characterized for its *in vivo* behavior regarding enhancement of the drug bioavailability.

## Materials and methods

### Materials

Agomelatine was kindly gifted by Hikma Pharma Co., Cairo, Egypt. Capryol 90^®^, Lauroglycol 90^®^, Labrafac Lipophile WL^®^, Labrafac CC^®^, Labrafil M 11944 Cs^®^, Labrasol^®^, Transcutol HP^®^, Plurol diisostearique^®^ were obtained as a gift from Gattefosse Co., Saint-Priest, France. Squalene, castor oil, isopropyl alcohol, isopropyl myristate (IPM), Cremophor EL^®^ and Cremophor RH40^®^ were purchased from Sigma-Aldrich Co., St. Louis, MO. Carbopol Ultrez 21^®^ was purchased from Lubrizol Co., Wickliffe, OH. Tweens, spans and propylene glycol were purchased from El-Nasr Pharmaceutical Chemical Co., Cairo, Egypt. All other chemicals and solvents were of analytical grade and used without further purification.

### Screening of oils, surfactants and cosurfactants

#### Screening of oils

For poorly soluble drugs, the loading of drug per formulation affects the total weight of formula used in delivering the therapeutic dose of drug (Azeem et al., 2009b). To choose the oil with the highest solubilizing capacity for agomelatine, the saturation solubility of agomelatine in different oils, such as Capryol 90, Lauroglycol 90, Squalene, Castor oil, IPM, Labrafil M1944 Cs was performed. Excess agomelatine was added to 2 mL of various oils, mixed with vortex mixer and then kept in shaking water bath at temperature 25 ± 0.5 °C for 72 h. Dispersions were centrifuged at 4000 rpm for 10 min and the agomelatine concentration was measured in the supernatant using UV–VIS spectrophotometer (UV-1601, Shimadzu, Kyoto, Japan) after suitable dilution with ethanol at *ʎ*_max_ 276.6 nm. Diluted solutions of oils were taken as blank. The oil with the highest solubilizing capacity for agomelatine was selected for further studies (Barot et al., 2012).

#### Screening of surfactants

The surfactant for developing agomelatine MEs was selected based on its solubilizing capacity for the selected oil. Briefly, aliquots of 10 µL of oil were added to 2.5 mL of 15% (w/w) aqueous solution of surfactant with vigorous vortexing till the appearance of turbidity. The solubility was determined using the following equation (Georgeta et al., 2015):

(1) $$Solubility\;of\;oil\;(\%w/w)=\frac{vd}{Q}.100$$

where *v* represents the volume (mL) of the selected oil added till the appearance of the turbidity, *d* is the density of the selected oil (g/mL) and *Q* is the quantity of surfactant contained in 2.5 mL of 15% (w/w) aqueous solution of surfactant.

#### Screening of cosurfactants

Choice of the cosurfactant was performed based on its ability to form the biggest ME region. The selected surfactant was mixed with 4 types of cosurfactants (Transcutol HP, propylene glycol, span 80 and Plurol diisostearique). At S_mix_ ratio of 1:1 w/w, the pseudoternary phase diagrams were plotted using the weight ratios of oil, S_mix_ as follow: 90:10, 80:20, 70:30, 60:40, 50:50, 40:60, 30:70, 20:80 and 10:90 w/w. The ME components percentages were then calculated and the pseudoternary phase diagrams were constructed. The transparent ME areas were determined.

#### *Selection of the optimum S*_mix_ *ratio*

Titration method was used to construct pseudoternary phase diagrams to select the most suitable S_mix_ ratio having the largest ME area (Barot et al., 2012). Altered ratios of S_mix_ (1:1, 1:2 and 2:1) were prepared. Then, the oil was mixed with these mixtures to give the weight ratios of 10:90, 20:80, 30:70, 40:60, 50:50, 60:40, 70:30, 80:20 and 90:10 w/w. These mixtures were titrated with distilled water drop wise while being magnetically stirred at ambient temperature. The mixtures were examined for clarity after each addition. The titration was continued until the solutions became cloudy or turbid. The quantity of water which made the mixtures turbid was recorded (Barot et al., 2012).

### Design and preparation of the ME formulations

D-optimal mixture experimental study was designed based on the three components, the selected oil (X_1_), the selected S_mix_ (X_2_) and water (X_3_). The range of each ME component was selected, based on the previous results obtained from the pseudoternary phase diagrams, as follows: The oil ranged from 5 to 10% and the S_mix_ was in the range of 30–55%. The highest percentages of water (40–60%), able to form ME with the remaining components, were adopted to increase the hydration of stratum corneum layer and so, facilitate the drug permeation. A group of candidate points were chosen by the software and this resulted in 11 formulations with five replicates, as shown in Table 1. The study was designed using Design-Expert software version 7 (Stat-Ease, Inc., Minneapolis, MN).

**Table 1.** The composition of ME formulations based on the D-optimal mixture design and the measured characteristics.

F	X_1_: oil	X_2_: S_mix_	X_3_: Water	*Y*_1_: GS (nm)	PDI	ZP (mV)	*Y*_2_: Optical clarity	*Y*_3_: Q_1_ (mg/cm^2^)	*Y*_4_: Q_24_ (mg/cm^2^)	*Y*_5_: ER
F1	5	35	60	34.0	0.38	−20.1	0.039	0.255	4.9	15.17
	5	35	60	33.6	0.32	−24.4	0.025	0.260	5.0	30.82
F2	5	45	50	46.8	0.26	−19.7	0.012	0.580	5.0	57.78
F3	5	55	40	42.8	0.33	−16.4	0.015	0.009	1.2	3.26
	5	55	40	28.9	0.33	−22.1	0.010	0.001	1.0	3.21
F4	6.25	38.75	55	36.4	0.23	−20.0	0.006	0.031	4.7	2.34
F5	6.25	48.75	45	26.3	0.29	−16.2	0.005	0.015	1.0	0.78
F6	7.5	32.5	60	19.1	0.32	−12.8	0.007	0.000	1.2	0.69
	7.5	32.5	60	32.3	0.20	−21.7	0.009	0.000	0.9	0.30
F7	7.5	42.5	50	42.6	0.20	−20.0	0.005	0.012	3.4	14.80
F8	8.75	36.25	55	25.1	0.26	−25.7	0.006	0.005	4.4	14.70
F9	10	30	60	37.1	0.25	−25.5	0.008	0.008	3.3	2.04
	10	30	60	25.0	0.32	−14.9	0.008	0.008	3.0	15.21
F10	10	40	50	21.3	0.22	−14.2	0.008	0.005	2.8	0.26
F11	10	50	40	16.0	0.13	−14.7	0.007	0.036	0.6	0.65
	10	50	40	15.8	0.19	−13.8	0.007	0.032	0.6	0.56

The surfactant and cosurfactant with the selected S_mix_ ratio were mixed with the oil in different proportions and the resultant mixtures were vortexed (JULABO Labortechnik, Seelbach, Germany) at ambient temperature. The drug was dissolved in these mixtures followed by the addition of the predetermined amount of distilled water.

### Evaluation of the prepared MEs

#### Determination of globule size (GS), polydispersity index (PDI), zeta potential (ZP) and optical clarity

Development of ME formulations with the minimal GS was a critical target for enhancing the transdermal permeation. On the other hand, PDI and ZP were considered as indicators for the particle size variability and the system physical stability, respectively. The GS, PDI and ZP of agomelatine loaded MEs were measured using Malvern Zetasizer (Zetasizer Nano ZS-90, Malvern instruments, Worcestershire, United Kingdom). Finally, the optical clarity of the prepared ME formulations was measured spectrophotometrically at 400 nm, using distilled water as a blank. Three samples were taken from each formula and analyzed and the average values ± standard deviation were recorded.

#### *Ex vivo* permeation

The *ex vivo* study was approved by Research Ethics Committee, Faculty of pharmacy, Cairo university, PI 1456. Skin samples were obtained from scarified newly born albino Wistar rats, and then examined for being intact without any cut or holes. After that, every sample was wrapped in aluminum foil, placed in polyethylene bags and stored in deep freezer at −20 °C till further use. To bring the skin pieces to room temperature before starting the permeation study, they were soaked in phosphate buffered saline (pH 7.4) at room temperature for 1 h (Wagner et al., 2000). The rat skin was clamped between the donor and the receptor chambers of modified Franz diffusion cells (area = 0.95 cm^2^), where the stratum corneum side faced the donor compartment and the dermal side faced the receptor compartment. The receptor compartment was filled with 10 mL 50% v/v ethanoic phosphate buffer saline (pH 7.4) to maintain sink conditions for agomelatine (saturated solubility = 0.5 mg/mL) (Magnusson & Koskinen, 2000; Raza et al., 2013b). The receptor chambers were thermostatically heated to 37 ± 0.5 °C and their content was magnetically stirred at 100 rpm through the whole experiment time. Each ME formulation (500 mg) containing 5 mg agomelatine was placed in the donor chamber. At time intervals of 0.5, 1, 2, 4, 6, 8 and 24 h, all the receptor chamber solution was withdrawn and immediately replaced with equal volume of fresh medium. The concentration of agomelatine in the withdrawn samples was determined using HPLC (Shimadzu, Kyoto, Japan) equipped with an isocratic pump and a reversed phase C18 column (3.9 × 300 mm, particle size 5 µm; Waters, MA) at *ʎ*_max_ of 230 nm. A mixture of 50:50 v/v acetonitrile and potassium dihydrogen phosphate buffer (15 mMol) was used as a mobile phase (pH 3.5), running at a flow rate of 1.0 mL/min (Liu et al., 2013). The analysis method had been validated.

For each formulation, the cumulative amount permeated of agomelatine (mg/cm^2^) was plotted as a function of time (*t*). Drug flux at a steady state (J_ss_) was calculated by dividing the slope of the most linear part of the graph by the area of the employed diffusion cell. Enhancement ratio (ER) was calculated using the following equation (Xie et al., 2017):

(2) $$ER=\frac{{Formulation\;J}_{ss}}{{Control\;J}_{ss}}$$

Where the control formula was aqueous suspension equivalent to 5 mg agomelatine.

### Optimization of the ME formulations

The mean GS (Y_1_), optical clarity (Y_2_), cumulative amount permeated after 1 h (Q_1_, Y_3_), cumulative amount permeated after 24 h (Q_24_, Y_4_) and ER (Y_5_) were utilized as the traced responses (dependent variables). Linear, quadratic and special cubic models are the most appropriate models for mixture designs consisting of three components. The best model was selected based on higher values of adjusted *R*^2^ and predicted *R*^2^_._ Adjusted *R*^2^ and predicted *R*^2^ should be within 0.2 of each other to ensure the validity of the model. The term ‘Adequate precision’ indicates signal to noise ratio, and it is desirable to be more than 4 (Huang et al., 2004). The optimum formulation was selected to have the smallest GS, the highest optical clarity, cumulative amount permeated after 1 h (Q_1_), cumulative amount permeated after 24 h (Q_24_) and enhancement ratio (ER).

### Preparation and characterization of the ME gel formula

The optimum ME formula was converted into gel to improve the retention of formula on the skin. This was done by adding carbopol^®^ Ultrez 21 (0.2% w/w) into the optimized ME formula and it was left overnight to allow dissolution and swelling of the gelling agent followed by dropwise addition of tri-ethanolamine (0.3%). The prepared agomelatine ME gel formula was characterized through measuring its GS, optical clarity and *ex vivo* characteristics (Q_1_, Q_24_ and ER) in comparison with 0.2% w/w carbopol gel containing the same amount of the suspended drug (Agomelatine hydrogel).

Moreover, samples were taken from the ME gel formula and transferred into rheometer plate having a CPE-41 spindle (Brookfield viscometer HBDV-I, Middleboro, MA). The applied rotation per minute ranged from 2 to 100 keeping the % torque within the acceptable limits (Morsi et al., 2014). Viscosity and shear stress values were determined at each corresponding rate of shear. The power model was used to analyze and characterize the flow properties of the test formula.

(3) $$\tau =K\gamma^{n}$$

Where *τ* is the shear stress (dyne/cm^2^), *K* is the consistency index (dyne/cm^2^.s^n^), *γ* is the rate of shear (s^−1^) and *n* is the flow index. Flow index higher than unity could indicate Newtonian flow whereas shear-thinning flow is pinpointed if the value was less than 1. On the other hand, the flow index value could exceed the unity in case of shear thickening systems (Ye et al., 2017).

### Imaging by transmission electron microscope (TEM)

The optimized ME gel formula was examined using transmission electron microscope (JEM-1230, Jeol, Tokyo, Japan). Samples were taken from the formula and spread over a carbon coated copper grid. Then, phosphotungistic acid 2% w/v solution was utilized to stain the placed samples. Finally, samples were left to dry at room temperature and visualized at 100 kV.

### *In vivo* bioavailability of optimized ME gel formula

#### Study design

Nine white rabbits (weight ≈ 3–4 kg) were used in the study. The protocol of the study was reviewed and approved (PI 1456) by research ethics committee, Faculty of Pharmacy, Cairo University (REC-FOPCU). The rabbits were housed two per cage at room temperature with free access to food and water with a 12 h light–dark cycle. The dorsal hair was removed using hair removal cream to facilitate application of the formula to the skin, then the rabbits were divided into three groups. Three-way, three-period, crossover design was applied with one-week washout period. An equivalent dose of 1 mg from either the ME gel formula or the reference agomelatine hydrogel was applied on the dorsal skin of each animal of the 1st and 2nd groups, respectively. On the other hand, equivalent drug solution (1 mg/mL) was orally administered to the third group. The applied dose was calculated based on dose translation from animal to human studies (Reagan-Shaw et al., 2008). At time intervals 0.25, 0.5, 1.0, 1.5, 2.0, 2.5, 3.0, 4.0, 5.0, 6.0, 8.0 and 24.0 h following application, blood samples were withdrawn from the marginal ear vein after local anesthetic cream is applied on the collection site 10 min prior to sampling. The blood samples were collected in 2 mL vacutainer tubes containing EDTA and then centrifuged at 4000 rpm for 10 min. The supernatant was transferred into another PE tubes, sealed and stored at −20 °C until assayed.

#### Assay method

Agomelatine was analyzed in plasma samples using Triple Quadrupole LC/MS/MS Mass Spectrometer (Micromass, Manchester, United Kingdom). Plasma samples (0.5 mL) were placed in 7 mL glass tubes, and then 100 µL of internal standard solution (1.6 µg/mL Clonazepam) was added. Samples were then vortexed. The extraction solvent (4 mL ethyl acetate) was added then samples were vortexed for 1 min. Samples were then centrifuged at 4000 rpm for 10 min at 4 °C (Eppendorf centrifuge 5804 R, Hamburg, Germany). The organic layer was separated into clean Wassermann tubes and dried using vacuum concentrator (Eppendorf 5301, Hamburg, Germany). The dried residues were reconstituted through vortexing with 200 µL of the mobile phase for1 min. and finally, placed into the autosampler of the LC-MS/MS. Samples of 20 µL were injected into a Shimadzu Prominence (Shimadzu, Japan) series LC system equipped with degasser (DGU-20A3) using sunfire column (50 mm ×5 µm). The isocratic mobile phase (80% acetonitrile + 20% 0.01 M Ammonium formate) was delivered at a flow rate of 1.0 mL/min into the mass spectrometer’s electrospray ionization chamber. Quantitation was achieved by MS/MS detection in positive ion mode for both agomelatine and clonazepam (IS) using a MDS Sciex (Foster City, CA) API-3200 mass spectrometer, equipped with a Turbo Ionspray interface at 500 °C. The ion spray voltage was set at 5500 V. Detection of the ions was performed in the multiple reactions monitoring (MRM) mode, monitoring the transition of the m/z 244.03 precursor ion to the m/z 185.30 for agomelatine and m/z 315.96 precursor ion to the m/z 270.00 for the internal standard. The Q1 and Q3 quadrupoles were set on unit resolution. The analytical data were processed by Analyst software version 1.4.2 (AB Sciex Pte. Ltd., Woodlands, Singapore).

#### Pharmacokinetic parameters and statistical analysis

The mean concentrations of agomelatine in plasma were plotted against time. The peak plasma concentration (C_max_) as well as the time to reach this peak (*t*_max_) was determined for each employed animal. The areas under agomelatine concentration-time curve till last time (AUC_0–24 h_) and till infinity (AUC_0–∞_) were calculated using the trapezoidal method. Elimination half-life (*t*_1/2_) and mean residence time (MRT) were calculated using Kinetica software program version 4.4.1 (Thermo Fisher Scientific Inc., Waltham, MA). Results were expressed as mean values ± standard deviations. The obtained pharmacokinetic data were analyzed using SAS^®^ (SAS Inc., Cary, NC) university edition through the general linear model (GLM) to calculate the arithmetic means and standard deviation of all continuous variables. The utilized SAS code was as follows (Choi et al., 2014):

proc glm data = agomelatine;

class formulation subject period sequence;

model log**X**= sequence subject (sequence) period formulation;

estimate “test-ref” formulation −1 + 1;

test h = sequence e = subject(sequence);

lsmeans formulation/adjust = t pdiff = control(“R”) CL alpha = 0.10;

run;(4)

*Where X was entered as C_max_, AUC_0–24 h_ or AUC_0–∞_.*

## Results and discussion

### Screening of oils, surfactants and cosurfactants

#### Screening of oils

When ME is formulated using an oil having high drug solubilizing power, a lesser amount of oil could be used to dissolve the desired drug dose. Consequently, lower surfactant concentration will be needed to solubilize the oil and this could increase the safety and tolerability of the system (Georgeta et al., 2015). Capryol 90 showed the highest solubilizing power for agomelatine as demonstrated in Figure 1(A). It is a semi-synthetic medium chain derivative having surfactant properties (Constantinides, 1995). This could be considered as an added value supporting the selection of Capryol 90 as an oily phase for the development of ME formulation.

**Figure 1.** Screening of oils (A), surfactants (B) and cosurfactants (C), in addition to selection of the optimum Smix ratio (D).

#### Screening of surfactants

The surfactant selection is critical for the development of MEs, as it is an important factor for controlling the spontaneous formation of a stable ME formulation. The surfactants act by forming a film at the oil water interface, which leads to the reduction of interfacial tension and consequently spontaneous formation of MEs (Chen et al., 2004). It is crucial to select the surfactant with a proper HLB value but with a minimum necessary concentration. Nonionic surfactants were selected because of their safety, biocompatibility, high stability, low sensitivity to pH changes or the presence of electrolytes or charged molecules and biocompatible nature (Constantinides, 1995; Georgeta et al., 2015). In our study, selection of surfactant was governed by its solubilization efficiency for the selected oil phase. Cremophor RH40 showed the highest solubilizing efficiency for Capryol 90 as shown in Figure 1(B) and so, it was selected for further studies.

#### Screening of cosurfactants

Addition of cosurfactants leads to an additional reduction in the interfacial tension and increases the fluidity of surfactant layer, thus expanding the microemulsion area (Lawrence & Rees, 2012; Georgeta et al., 2015). The microemulsion area in the pseudo-ternary phase diagrams was used to evaluate the emulsification potential of the cosurfactants. Figure 1(C) presents the pseudoternary phase diagrams constructed for Capryol 90 (oil phase), water, Cremophor RH40 and four different cosurfactants (Transcutol HP, propylene glycol, span 80 and Plurol diisostearique) at a fixed S_mix_ ratio (1:1). Transcutol HP was chosen as the cosurfactant of choice for agomelatine MEs construction as it had shown the largest ME area in the ternary phase diagram.

#### *Selection of the optimum S*_mix_ *ratio*

Pseudo-ternary phase diagrams were plotted for the three selected S_mix_ ratios 1:1, 1:2 and 2:1 w/w surfactant to cosurfactant. Clear and stable MEs were obtained by the three S_mix_ ratios but the one which gave the largest area was 1:2 w/w, as illustrated in Figure 1(D). Therefore, this ratio was selected for further studies.

### Evaluation of the prepared MEs

#### Determination of globule size (GS), polydispersity index (PDI), zeta potential (ZP) and optical clarity

GS of the ME affects its stability, skin penetration and hence *in vivo* efficacy (Xi et al., 2009; Wang et al., 2012). As shown in Table 1, the GS of the various ME formulations ranged from 15.8 to 46.8 nm. Linear model was the most suitable one fitting the *Y*_1_ values (*p* value = .0335) with non-significant lack of fit (*p* value = .3789) and adequate precision of 5.3 indicating the model ability to navigate the design space with the minimal pure error (Elbary et al., 2011). ANOVA analysis on GS (nm) of ME (Y_1_) shows that linear mixture components have a significant effect on GS (*p* value < .05). Formula 11 which showed the smallest GS was composed of 10% oil, 50% S_mix_ and 40% water as illustrated in Figure 2(A). This may be due to the low content of water and high content of S_mix_ which allows more reduction of the interfacial tension, which results in better reduction of ME GS (Shah et al., 2009; Xi et al., 2009). Decreasing the GS could increase the contact surface area between the skin and the ME system, and so facilitate the drug transport across the skin (Khurana et al., 2013). The regression equation relating different factors and interactions for the GS in terms of coded variables was as follows:

(5) $$Y_{\text{1}}=-\text{35}.{\text{58X}}_{\text{1}}+\text{34}.{\text{54X}}_{\text{2}}+\text{39}.{\text{84X}}_{\text{3}}$$

**Figure 2.** Contour diagrams for the effect of formulation variables on the globule size (A), optical clarity (B), Q1 (C), Q24 (D), ER (E) and desirability (F).

As shown in Table 1, the PDI of various ME formulations varied between 0.13 and 0.38. This low PDI values indicated the uniformity of the GS within each formulation (Biruss et al., 2007). Moreover, the ZP values of various ME formulations varied between −12.8 and −25.7 mV indicating the reasonable physical stability of most ME formulations prepared (White et al., 2007).

The optical clarity of the different ME formulations ranged between 0.005 and 0.039 nm, as displayed in Table 1. The high optical clarity of MEs could indicate the effective emulsification of Capryol 90 into water which resulted in the formation of isotropic MEs (Date & Nagarsenker, 2008). The quadratic model adopted for the analysis of the obtained optical clarity values. It had been validated through its high adequate precision (9.775) and its non-significant lack of fit (*p* value = .5251). Factorial ANOVA of the optical clarity values showed that the linear mixture had a significant effect on the traced response values (*p* value = .0037) with significant interactions between oil/S_mix_ and oil/water percentages. It could be observed from Figure 2(B) that decreasing water with increasing the oil and the S_mix_ percentages could increase the optical clarity of the prepared ME formulations. The regression equation describing the effect of different factors of the traced response was as follows:

(6) $$Y_{\text{2}}=0.{\text{78X}}_{\text{1}}+0.0{\text{11X}}_{\text{2}}+0.0{\text{38X}}_{\text{3}}-0.{\text{99 X}}_{\text{1}}{\text{X}}_{\text{2}}-\text{1}.{\text{11X}}_{\text{1}}{\text{X}}_{\text{3}}-0.0\text{2}0{\text{ X}}_{\text{2}}{\text{X}}_{\text{3}}$$

#### *Ex vivo* permeation

As shown in Table 1, the Q_1_ of the various ME formulations varied between zero and 0.580 mg/cm^2^, the Q_24_ of different ME formulations ranged from 0.6 to 5.0 mg/cm^2^ and the ER of the various ME formulations varied between 0.26 and 57.78. The cubic model was the most fitting one to the values of three responses Q_1_ (Y_3_), Q_24_ (Y_4_) and ER (Y_5_). The lack of fit was non-significant relative to the pure error (*p* value > .05) with high adequate precision (> 4) in each of the three responses indicating the adequate signal to noise ratio (Barton, 2013). The factorial equations correlating the studied factors to the measured responses were as follow:

(7) $$Y_{\text{3}}=-\text{194}.0{\text{8X}}_{\text{1}}\text{+5}.{\text{298}}^{-\text{3}}{\text{X}}_{\text{2}}+\;0.{\text{23X}}_{\text{3}}+\text{ 338}.0{\text{6X}}_{\text{1}}{\text{X}}_{\text{2}}+\text{ 322}.{\text{44X}}_{\text{1}}{\text{X}}_{\text{3}}+\text{ 1}.{\text{63X}}_{\text{2}}{\text{X}}_{\text{3}}-\text{ 3}0\text{2}.{\text{32X}}_{\text{1}}{\text{X}}_{\text{2}}{\text{X}}_{\text{3}}+\text{158}.{\text{79X}}_{\text{1}}{\text{X}}_{\text{2}}\left({\text{X}}_{\text{1}}-{\text{X}}_{\text{2}}\right)\;+\text{ 134}.{\text{88X}}_{\text{1}}{\text{X}}_{\text{3}}\left({\text{X}}_{\text{1}}-{\text{X}}_{\text{3}}\right)\;+\text{ 1}.{\text{95X}}_{\text{2}}{\text{X}}_{\text{3}}\left({\text{X}}_{\text{2}}-{\text{X}}_{\text{3}}\right)$$

(8) $$Y_{\text{4}}=-\text{1}0\text{5}0.{\text{66X}}_{\text{1}}+\text{1}.0{\text{8X}}_{\text{2}}–{\text{ 5X}}_{\text{3}}+\text{17}0\text{1}.{\text{96X}}_{\text{1}}{\text{X}}_{\text{2}}+\text{ 1882}.{\text{85X}}_{\text{1}}{\text{X}}_{\text{3}}+\text{33}.\text{5}0{\text{ X}}_{\text{2}}{\text{X}}_{\text{3}}-\text{ 1661}.{\text{18X}}_{\text{1}}{\text{X}}_{\text{2}}{\text{X}}_{\text{3}}+\text{65}0.{\text{86X}}_{\text{1}}{\text{X}}_{\text{2}}\left({\text{X}}_{\text{1}}-{\text{X}}_{\text{2}}\right)+\text{873}.{\text{96X}}_{\text{1}}{\text{X}}_{\text{3}}\left({\text{X}}_{\text{1}}-{\text{X}}_{\text{3}}\right)\;-\text{ 35}.{\text{15X}}_{\text{2}}{\text{X}}_{\text{3}}\left({\text{X}}_{\text{2}}-{\text{X}}_{\text{3}}\right)$$

(9) $$Y_{\text{5}}=-\text{2}0\text{52}.{\text{56X}}_{\text{1}}+0.{\text{48X}}_{\text{2}}\text{-2}.0{\text{2X}}_{\text{3}}+\text{ 3355}.0{\text{7X}}_{\text{1}}{\text{X}}_{\text{2}}+\text{ 347}0.{\text{89X}}_{\text{1}}{\text{X}}_{\text{3}}+\text{ 11}.{\text{6X}}_{\text{2}}{\text{X}}_{\text{3}}-\text{ 289}0.{\text{31X}}_{\text{1}}{\text{X}}_{\text{2}}{\text{X}}_{\text{3}}+\text{1321}.\text{9}0{\text{X}}_{\text{1}}{\text{X}}_{\text{2}}\left({\text{X}}_{\text{1}}-{\text{X}}_{\text{2}}\right)+\text{1484}.{\text{34X}}_{\text{1}}{\text{X}}_{\text{3}}\left({\text{X}}_{\text{1}}-{\text{X}}_{\text{3}}\right)-\text{1}0.{\text{44X}}_{\text{2}}{\text{X}}_{\text{3}}\left({\text{X}}_{\text{2}}-{\text{X}}_{\text{3}}\right)$$

ANOVA analysis on Q_1_ (Y_3_), Q_24_ (Y_4_) and ER (Y_5_) of MEs showed that the linear mixture was significant (*p* value < .05) with significant interactions between each of the three components, i.e. oil, water and S_mix_. It could be noticed from Figure 2(C–E) that decreasing the oil and increasing the S_mix_ could increase Q_1_, Q_24_ and ER. Decreasing oil percentages could minimize the affinity of agomelatine as a lipophilic drug to remain in the ME phase and enforce its partitioning to the stratum corneum (Yuan et al., 2006). Moreover, increasing S_mix_ content could facilitate the fluidization of the lipid bilayer within skin and so, support the drug permeation into the systemic circulation (Hua et al., 2004).

### Selection of the optimized ME formulation

The aim of the optimization of pharmaceutical formulations was to obtain a high quality system based on the predetermined levels of variables (Basalious et al., 2010). A numeric analysis was used to select the optimum formula using the design expert software. Figure 2(F) shows an optimum region which covered the requirement of the traced responses. Based on the selection criteria, MEs which have the smallest GS optical clarity, and the highest Q_1_, Q_24_ and ER were chosen. Upon assessment of the available solutions, desirability function was used to select the optimum composition. A ME formulation satisfying these criteria with a desirability of 0.868 had X_1_, X_2_ and X_3_ values of 5, 45 and 50%, respectively, which was the composition of formula F2 already employed in the design. The ME formula with the optimum composition had been prepared to be subjected to further processing and characterization.

**Figure 3.** Rheological (A) and morphological (B) characteristics of the optimized ME gel formula.

### Characterization of the ME gel formula

Globule size (35.82 nm) and optical clarity (0.012 nm) of the optimized formula had not been significantly altered after gelling (*p* value > .05). Significant enhancement of permeation was observed in case of the optimum ME gel relative to the drug suspended in carbopol gel, as demonstrated in Figure 4(A), with Q_1_, Q_24_ and ER of 0.4, 4.5 mg/cm^2^ and 37.30, respectively. This might be due to the nano-size of the optimum formulation in addition to the presence of surfactant and cosurfactant which might lead to a significant disruption of the lipid bilayer present in the stratum corneum (Ustundag Okur et al., 2017). Regarding the rheological characteristics, viscosity of the ME gel formula decreased upon increasing rate of shear, as shown in Figure 3(A). This was confirmed through the very low value of the flow index (0.0681) which revealed the shear thinning behavior of the investigated gel. This could be beneficial for physical stability of the dispersion minimizing the possibility of globule aggregation and size growth during storage. Furthermore, the decreased viscosity with rubbing could facilitate spreading of the applied gel to form a thin layer on the skin. Finally, viscosity would increase again after application keeping the drug in contact with the skin for longer time and sustaining the drug release from the globules (Abdelrahman et al., 2015).

**Figure 4.** *Ex vivo* (A) and *in vivo* (B) permeation profiles of optimized ME gel in comparison with the drug hydrogel and the oral drug solution.

### Imaging by transmission electron microscope (TEM)

TEM imaging shows the ME gel globules in the range of 27–38 nm, as shown in Figure 3(B), going in harmony with the Z-average measured by Zetasizer. The imaged globules were almost spherical with smooth surface. There was no observed aggregation indicating a good dispersibility of the ME globules. This might be referred to the reasonable ZP on the globules surfaces (Dehghani et al., 2017).

### *In vivo* bioavailability of optimized ME gel formula

The mean agomelatine concentrations in rabbits’ plasma after administration of the optimum ME gel formula, agomelatine hydrogel and oral solution (reference) are displayed in Figure 4(B). The optimum ME gel formula was found to have higher C_max_, AUC_0–24  h_, AUC_0–∞_ than the agomelatine hydrogel and oral solution, as shown in Table 2. These data were analyzed using SAS software (SAS Inc., Cary, NC) and the output indicates the significance difference between the test and the reference hydrogel in aspects of the AUC_0–24 h_, AUC_0–∞_ with *p* values of .0493 and .0146, respectively. On the other hand, the C_max_ difference was non-significant between the two formulations (*p* value = .0839). Furthermore, the point estimates calculated for the C_max_, AUC_0–24 h_ and AUC_0–∞_ were 236.41, 213.99 and 245.15%, respectively. These obtained findings could emphasize the superior ability of the optimized ME gel over the reference hydrogel to enhance the agomelatine transdermal permeability. On the other hand, oral agomelatine solution showed significantly lower C_max_, AUC_0–24 h_ and AUC_0–∞_ than the transdermally applied either ME gel or hydrogel. This could be referred to the previously stated extensive 1st pass metabolism limiting the absolute bioavailability of oral agomelatine to be 5% only (Du et al., 2013). Moreover, the elimination half-life and the MRT of the optimal ME gel formula was significantly higher than the reference hydrogel (*p* value < .0001) indicating the sustainment of the drug permeation all over the experiment time (Elshafeey et al., 2009).

**Table 2.** Pharmacokinetic parameters of the optimized ME gel formula in comparison with the drug hydrogel and oral solution (A) and SAS analysis of C_max_, AUC_0–24 h_ and AUC_0–∞_ (B).

(A)				
	Treatment (mean ± SD)			
Pharmacokinetics parameters	Optimized ME gel	Drug hydrogel	Oral drug solution	
C_max_ (ng/mL)	122.00 ± 99.32	43.85 ± 20.61	24.68 ± 8.56	
T_max_ (h)	1.13 ± 0.80	1.50 ± 2.04	0.5 ± 0.00	
AUC_0–24 h_ (ng.h/mL)	270.02 ± 104.56	135.33 ± 71.77	59.67 ± 12.57	
AUC_0–∞_ (ng.h/mL)	332.91 ± 139.92	145.28 ± 74.08	92.99 ± 21.05	
K_e_ (l/h)	0.11 ± 0.04	0.22 ± 0.06	0.04 ± 0.00	
t_½_ (h)	7.24 ± 2.34	3.37 ± 0.87	17.88 ± 1.48	
MRT (h)	12.62 ± 5.15	8.61 ± 3.11	22.49 ± 4.20	
(B)				
C_max_				
DF	1	4	1	1
Type III SS	0.31647282	0.27094836	2.76440032	2.22093451
Mean square	0.31647282	0.06773709	2.76440032	2.22093451
F value	0.75	0.16	6.53	5.24
Pr > F	0.4361	0.9482	0.063	0.0839
AUC_0–24 h_				
DF	1	4	1	1
Type III SS	0.09975565	1.19820373	0.23013033	1.73642523
Mean square	0.09975565	0.29955093	0.23013033	1.73642523
F value	0.45	1.34	1.03	7.78
Pr > F	0.5403	0.3911	0.3673	0.0493
AUC_0–∞_				
DF	1	4	1	1
Type III SS	0.08532882	1.35585856	0.42233766	2.41223985
Mean square	0.08532882	0.33896464	0.42233766	2.41223985
F value	0.6	2.38	2.97	16.97
Pr > F	0.4817	0.2103	0.1599	0.0146

## Conclusions

In this study, ME components were screened and selected based on a stepwise pyramidal screening to ensure the selection of the most suitable oil, surfactant and cosurfactant for the incorporated drug. D-optimal mixture design was applied to obtain the optimal agomelatine loaded ME composition having the smallest GS and the highest optical clarity Q_1_, Q_24_ and ER. The optimized ME formulation was composed of 5% oil, 45% S_mix_ (Cremophor RH40: Transcutol HP in ratio 1:2 w/w), 50% water. *Ex vivo* and *in vivo* permeation results could highlight that the optimized ME gel formula could be considered as a promising carrier for the transdermal delivery of agomelatine.
